# Football Game Video Analysis Method with Deep Learning

**DOI:** 10.1155/2022/3284156

**Published:** 2022-06-08

**Authors:** Nian Liu, Lu Liu, Zengjun Sun

**Affiliations:** ^1^Department of Sports, Zhejiang Gongshang University, Hangzhou 310000, Zhejiang, China; ^2^Business & Public Administration, Namseoul University, Cheonan 31020, Republic of Korea

## Abstract

Football is a beloved sport, and its wide audience makes football video one of the most analytically valuable types of video. Researchers have achieved certain research results in football video content analysis. How to locate interesting event clips from a complete long video is an urgent issue to be addressed in football game video analysis. The granularity of sports event detection results with traditional machine learning is relatively coarse, and the types of events that can be detected are limited. In recent years, deep learning has made good progress in the research of video single-person events and action detection, but there are few achievements in the detection of sports video events. In response to this problem, this work uses a deep learning method to build an event detection model to detect events contained in football videos. The whole model is divided into two stages, in which the first stage is utilized to generate candidate event fragments. It divides the football video to be detected into a sequence of frames of a certain length and scans using a sliding window. Multiple frame sequences within a sliding window form a segment, and each segment is a prediction unit. The frame sequence features within the segment are obtained through a three-dimensional convolutional neural network, which is used as the input of each time point of the bidirectional recurrent neural network and further integrated to generate the event prediction of the segment. The second stage is to further process the above results to remove all segments predicted as nonevents. The thresholds are set according to the detection effect of various events to filter out event fragments with higher probability values, obtain the start and end positions of the events through merging, classify and mark them, and finally output complete event fragments. This work has carried out comprehensive and systematic experiments to verify correctness of the proposed method.

## 1. Introduction

People's production and lifestyle have undergone tremendous changes. Traditional information media, such as books, documents, newspapers, records, movies, and TV programs, are increasingly appearing in people's daily life in digital form. Compared with other information sources, video has the characteristics of intuition and large amount of information and occupies a large share in practical applications. While bringing a rich audio-visual experience, the rapid expansion of the number of digital videos has also made the problem of insufficient video processing capacity more prominent, posing new challenges to the management, editing, and distribution of digital media. How to intelligently analyze the content of video clips through a computer, so as to automatically retrieve and locate relevant video clips through a computer according to user requirements, has become an urgent issue to be solved in industry and academia. As a result, video content analysis technology has gradually become one of the current research hotspots with important theoretical and practical significance [1–5].

Researchers are trying to figure out how low-level features can be mapped to higher-level semantics so that users may get more convenient content acquisition services from video analysis technologies, which is the primary purpose of the research. There is a wide variety of video content, and the content found in videos from various professions varies greatly. Since video content analysis technology cannot be universal, an appropriate identification procedure must be devised based on the examined content's features. Football video has a huge fan base and a lot of money riding on it, so researchers have flocked to it because of the wealth of data it provides for content analysis. Football video content analysis is in high demand since football fans want to view only the most relevant clips, such as highlights and key moments. Many football fans and professionals want an easy way to rapidly find specific attack types among a big number of assault footage. In order to better comprehend the gaming process and achieve better results, these users anticipate to evaluate the techniques and tactics used in past games. Football video strategy and tactical analysis research is sparse, and the relevant needs have not been fully satisfied [6–10].

Football video event detection has gradually become an important research content in the current sports video analysis field, as illustrated in Figure 1. When detecting events in sports videos based on the traditional machine learning methods, the low-level features of the videos are mainly extracted.

However, the color of the football video itself is relatively simple, and the events mainly occur in the medium and long shots. The appearance outline of some things is difficult to accurately capture, so it cannot show a good detection effect. Later, an artificial mechanism was added, using human prior knowledge and established rules to assist. Although this improves the detection performance to a certain extent, because the rules are relatively simple, it cannot fully express the relationship between objects and people's cognitive emotions. The quality of the detection results largely depends on human experience, and the scalability of the model is poor. Based on the successful application of semantic analysis in the field of artificial intelligence, some scholars have further introduced it into the field of video analysis. From the perspective of visual understanding, the original data in the video are abstracted into a concept that conforms to human vision. The idea of semantic analysis is the same as people's habit of cognition of things. The semantic expression of video is the deep interpretation of video content by people. The emergence of deep learning has enabled videos to achieve better results in semantic analysis. Deep learning has made significant progress in image recognition, video analysis, and other fields. It is a neural network that can simulate human learning behavior. By constructing a multilayer model and using a large amount of data for training, it can automatically learn more useful features, which can fully express the internal information of video data. Deep learning is an important branch [11–15].

The purpose of this research is to analyze the semantic features in football videos and use the deep learning method to complete the event detection and classification of football match videos. The main work includes the following aspects: (1) event classification, using the convolutional neural network to extract features from existing video clip sequences, including global features and local features. By further integrating the features, the event type to which the segment belongs is predicted. (2) Event detection, adding a recurrent neural network with a classification network to further learn sequence features and determine the time boundary of the event. Then, by filtering and merging fragments containing events, complete events of different lengths are obtained and types are marked.

## 2. Related Work

Reference [16] used CNN to separately extract features from images of video frames and integrate features of all frames to form video descriptors. It concatenated the video's RGB descriptor and optical flow descriptor to form a video descriptor. Reference [17] proposed a three-dimensional convolution method that could convolve from the space of the video image and the time of the frame sequence at the same time. By concatenating multiple convolution layers and downsampling layers to form an action recognition network, it had achieved good results in human action recognition in surveillance videos. Reference [18] also proposed a 3D convolution method, which could be well integrated with 2D convolution network to form a C3D network. Reference [19] proposed a network structure that can perform feature extraction in spatial and temporal information of video. Different from the above two kinds of 3DCNNs that performed convolution in space and time at the same time, this method separated the convolution in space and space, first convolving in space, and then convolving in time dimension. Reference [20] utilized 2D CNN as well as 3D CNN to integrate features of different granularities on video frame sequences and then combined LSTM for action recognition. References [21, 22] used 2D convolution and 3D convolution to process video images and fused two branches at fully connected layer to obtain action type. In reference [23], a new network convolution method was proposed, which made the image feature sequence and optical flow image sequence better fuse and realized the end-to-end training of the network. Reference [24] fine-tuned the existing CNN model and only fused all the frames of the video through the maximum pooling layer at the end to obtain the description features of the video. Reference [25] used Fisher vector or VLAD encoding to further re-encode the video features extracted by CNN, which made the feature utilization more efficient. In reference [26], in addition to using FC features, features of multiple convolutional layers in the middle of the network were also used to construct video features. Reference [27] used CNN to extract features of original frame image and optical flow image respectively, obtained the image features and optical flow features of the entire video through pooling operation, and used LSTM to process the two features respectively. Then, it combined the results of the two to-do video classification. Reference [28] also combined CNN and multilayer LSTM for video event analysis and set the output of LSTM as text, so that the model could finally generate a simple text description of the video.

Reference [29] used multibox to detect the player's position area in the video frame for the basketball game video and then used the inception network to extract the video frame and the features of each player respectively. It used BLSTM to process the frame sequence and player feature sequence respectively and used the output of these two networks as input to construct an event recognition LSTM. Reference [30] also combined CNN and LSTM to detect volleyball video events, used CNN to extract player features, and built LSTM network for each player separately. The output of the single-person LSTM was pooled to obtain the overall state, and the LSTM was constructed based on this input to identify the overall activity state of the team. Reference [31] combined CNN and RNN-based visual attention models to focus visual attention on keyframes for event prediction. It used reinforcement learning to train the model, enabling the system to automatically learn during the interaction with the video image sequence, and directly output the time boundary of the action. The next step of the localization model should focus on the processed video frames. The research object of reference [32] was the first-person motion video, and they used two CNN network structures to process the video at the same time. One was a traditional 2D CNN that analyzes the spatial static features of video frames. The other was 3D CNN, which analyzed dynamic features in the temporal dimension of video frame sequences. A sorting algorithm was proposed to sort the outputs of the two networks and select the highlights in the video. Reference [33] improved the C3D network, so that the convolution step size of the network in the time dimension could be adjusted according to the needs, and based on this, three networks with different functions of preselection, classification, and positioning were constructed to locate the action time boundary. Reference [34] fused DT and CNN features of frame images and used a fixed-length sliding window to sequentially process the video to obtain the detection results of action clips. References [35, 36] proposed a method of extracting and integrating the dynamic features of video clips in multiple temporal widths, centered on a certain frame, and combining RNN to detect action temporal boundaries. An action detection problem had been solved utilizing a new CNN structure that uses CNN to identify the action type and the sliding window to identify the boundary. In reference [37], the action detection network used C3D and a longer RNN as the core model of the action detection network and predicted time boundaries based on output hidden states of the RNN. In addition, different lengths of predictions were generated for each forecast. Although the boundary was predicted with RNN, although the boundary determination of the sliding window is avoided in the detection process, the longer RNN network structure was deeper. During the learning process, problems such as gradient disappearance and difficulty in parameter learning were prone to occur, which affected the final detection result.

## 3. Football Events Classification

Event classification is one of the research contents of event detection, and accurate classification of events can improve the effect of event detection to a certain extent. The most important thing in classification is to obtain effective information about events, so how to learn and describe event features are the main research contents of this section. Using deep learning methods, two-dimensional convolutional networks and three-dimensional convolutional networks are used to extract features from events.

### 3.1. Feature Extraction

Feature extraction is one of the important research issues in the field of video analysis. The traditional hand-designed features are relatively independent and cannot represent the deep content of the video well. Deep learning adopts a multilayer learning method, which can automatically learn features from big data and combine them to form a more effective expression. The most important thing in deep learning is feature learning. Therefore, the reasonable selection of models for feature extraction and description plays an important role in the effect of event classification. Since the application of convolutional neural networks to handwritten digit recognition, CNN has made significant progress in the field of image recognition, and a series of improved models have emerged. Compared with other models, when GoogLeNet achieves better classification results, it uses fewer hierarchical structures and requires a relatively small scale of parameters. Therefore, this section adopts Inception v2 from GoogLeNet as a candidate model for 2D convolutional networks. The basic structure of Inception v2 is the inception module, as shown in Figure 2.

Different from the traditional method of directly stacking convolutional layers, Inception v2 is composed of multiple inception modules. Two kinds of filters such as 1 × 1 and 3 × 3 are used in each module. This structure increases the width and depth of the network without increasing the computational load. In addition, the 5 × 5 convolution kernel in Inception v1 is replaced with two 3 × 3 convolution kernels, which reduces the number of parameters and improves the calculation speed, while ensuring the same number of features. Another improvement is to parallelize a 3 × 3 pooling operation with convolution to reduce feature loss caused by pooling when compressing features. In order to solve the problem that the input distribution also changes when the neural network is iterated due to parameter update during the training process, Inception v2 normalizes the input data before each layer is input. This avoids additional computational overhead for relearning different distributions and speeds up neural network training.

Although CNN has an excellent performance in image recognition, there are certain problems when it is introduced into the field of video analysis. There is a large correlation between the front and rear frames in the video, and when CNN processes video frames, it generally extracts features for each frame of image separately. This convolution method does not take into account the interframe motion in the time dimension, and it is easy to ignore the relevant information between frames. The frame processing process of 3D CNN is similar to that of CNN, and the differences are that it adds a time dimension to CNN and can extract features of multiple frame images at the same time. When extracting video sequence features, it is possible to save the motion state changes between the frames before and after, thereby improving the accuracy of event classification. Therefore, this section adopts 3D CNN as a candidate model for 3D convolutional networks. When 3D CNN is used to extract features from a video frame sequence, the frame sequence can be regarded as a cube. It is convolved with a 3D convolution kernel, which captures the motion information of the video. Since the convolution kernel weights of each layer are shared throughout the convolution process, only one type of feature can be extracted. When multiple features are required, multiple convolution kernels can be set.

### 3.2. Event Classification Model

The event classification model combines a 3D CNN and a Softmax classifier, as illustrated in Figure 3. The input is an event segment, and the sequence features are extracted from the original frame image through 3D CNN. The probability value is calculated using the Softmax classifier to get the predicted classification of the event.

The 3D CNN consists of a convolution layer, activation function, pooling layer, fully connected layer, and dropout layer. The specific network structure is shown in Figure 4. The input is split into two parts: the full-frame image and the central area of the frame. This is because the camera always places the current important moving scene in the center of the camera during the shooting process. Therefore, the probability of occurrence of events in this part is higher, and it is easier to capture the characteristics of events. The central area of the frame is half the size of the full frame.

Convolutional layers are used to extract features from consecutive frame sequences. Each layer uses a smaller convolution kernel to locally sense the input. In this way, each neuron in a convolutional layer only needs to connect local adjacent regions of the input unit, extracting local information. Global information can then be obtained by integrating at a high level. Compared with the traditional full connection method, more redundant information will not be generated, thereby reducing the complexity of network computing. In addition, the convolution kernel parameters of each layer are shared to reduce the number of parameters and improve the efficiency of feature extraction.

The output of the convolutional layer is a linear function, while in reality, it deals with more nonlinear problems. Therefore, an activation function is added to convert a linear function into a nonlinear function, so that the neural network has the ability to learn nonlinearly and solve more complex problems. The feature map output by the convolutional layer will maintain the same size as the original input, so a pooling layer is set after each convolutional layer to downsample the feature output of the convolutional layer. After the local features are extracted, the features need to be further integrated to obtain global information. The fully connected layer adopts a fully connected method to connect all neurons to each node of the previous layer, which can fully learn all features and classify them. However, the fully connected layer has many parameters, so only a two-layer structure is used.

The Softmax classifier is a generalization of logistic regression models for multiclassification problems. Since there are many different event types in this experiment, the Softmax classifier was chosen. The calculation method is as follows:

(1) $$\begin{array}{c} z_{e,c}=W_{c}f+b_{c},\\ p\left(y_{e}=c\right)=\frac{e^{z_{e,c}}}{\sum_{c=1}^{C}e^{z_{e,c}}}, \end{array}$$

where *y*_*e*_ is the event type predicted for event *e* and *p*(*y*_*e*_=*c*) is the probability value that event *e* is predicted to be class *c*.

### 3.3. Classification Model Training

The classification model is fine-tuned on the basis of the existing parameter model. Therefore, in the 3D CNN network, the existing parameter model is used as the initialization parameter, and the learning rate is 0.0001. The size of the convolution kernel of each convolutional layer is 3 × 3 × 3, and the sliding step size is 1 in both time and space. The pooling window size in the pooling layer is 2 × 2 × 2, and the sliding step size is 2. The dimensions of the output of each layer of the fully connected layer are 8192 and 4096 dimensions, respectively. When extracting features, 32 consecutive frames are randomly selected from each event segment, and a sliding window of size 16 is used to divide the 32-frame sequence into multiple subsequences. Each subsequence is used as an input to the model alone, with a sliding step size of 8. All parameters in the Softmax classifier are randomly initialized with an initial learning rate of 0.01.

A neural network with only convolutional layers is a simple linear regression model, and when the input is complex data types such as images, videos, and audio, it cannot fully learn the intrinsic properties of these data. Therefore, adding an activation function after the convolutional layer can realize the nonlinear function mapping of features to enhance the learning ability of the neural network. There are three choices of activation function: sigmoid function, tanh function, and ReLU function. Although the sigmoid function is easy to understand and apply, it has slow convergence and is prone to saturation. There will be a gradient disappearance problem during backpropagation, resulting in the parameters not being updated. The tanh function is improved on the basis of the sigmoid function, but there is also the problem of gradient disappearance. ReLU is a piecewise function, and when the function input is positive, it will keep the size of the value unchanged. When the input is negative, it becomes 0, making a subset of neurons in the neural network inactive to avoid overfitting the training set. In addition, since the ReLU function is a linear function in the non-negative interval and the gradient is equal, the problem of gradient disappearance is also avoided and the convergence speed of the model is guaranteed. Taken together, in the training of the classification model, the ReLU function is used as the activation function. The three activation function formulas are as follows:

(2) $$\begin{array}{c} \text{Sigmoid}\left(x\right)=\frac{1}{\left(1+\exp\left(-x\right)\right)},\\ \text{Tanh}\left(x\right)=\frac{\left(\exp\left(x\right)-\exp\left(-x\right)\right)}{\left(\exp\left(x\right)+\exp\left(-x\right)\right)},\\ \text{ReLU}\left(x\right)=\max\left(x,0\right), \end{array}$$

where *x* is the input feature.

Fine-tuning the existing parameter model can save a lot of training time. The most important thing in fine-tuning is to select the parameter tuning layer. In the experiment, the 3D CNN was trained by three schemes, and the training effects were compared. The first method is to fix the parameters of all layers unchanged. The second method is to fix all the parameters of the fully connected layer unchanged and fine-tune the parameters of other layers. The third method is to fine-tune the parameters of all layers.

## 4. Football Event Detection

Event detection is the process of locating the time boundary of an event in a complete football video and then classifying it. The event detection model designed in this section is based on the classification model and adds a time series feature integration module. In the model, the video is divided into frame sequences of a specific length, the entire video is scanned by a sliding window, and the starting position of the event is predicted by extracting and integrating the features of multiple frame sequences. The entire event detection process is shown in Figure 5.

### 4.1. Timing Feature Integration

Given that 3D CNN has achieved good results in event classification, when building an event detection model, 3D CNN is still used to extract features from frame sequences in videos. However, a complete football video is usually 45–50 minutes long and contains tens of thousands of frames, and the correlation between frames is relatively large. When only 3D CNN is used, the sequence length that can be processed is limited, and it is easy to ignore the dynamic information contained in the video. Therefore, in the event model, RNN is added to integrate the frame sequence features to further extract the event information contained in the video.

In the RNN network structure, nodes between hidden layers are fully connected. It adds the output of the hidden layer at the previous time point to the current input to realize the memory of the previous information. In this way, the correlation between the data before and after can be preserved, and the sequence data can be processed more efficiently. There are currently three popular RNN structures: traditional RNN, LSTM, and bidirectional recurrent network BRNN.

The hidden unit is the memory unit of the traditional RNN network. In addition to the input and output at each time point, it also receives the hidden state information from the previous time point and calculates it together with the current input. The emergence of traditional RNN networks has achieved great success in machine translation, image description generation, etc. but also has major shortcomings. When it is trained by the backpropagation algorithm, the RNN has a long time span and a deep level. The calculated gradient will show an exponential decrease or increase as the level increases, and the gradient will disappear or the gradient will explode, resulting in training failure. LSTM adds cell states and control gates to the traditional RNN structure. There are three control gates in the structure, which control whether the input, output, and hidden layer states are added to the unit state and the degree of influence on the unit state. In this way, the LSTM can selectively remember the key information it needs. Whether it is a traditional RNN network or an improved LSTM network, forward memory is used. In the video, what happens in the future has a strong correlation with the current state. In this regard, this section uses two layers of LSTM to form BLSTM to integrate sequence features, which can simultaneously access past and future contextual information.

### 4.2. Time Boundary Detection

The time for various football events to occur is generally 3 to 4 seconds, and they appear in any time period in the game video. Therefore, in event detection, the video is first divided into a sequence of frames of a certain length. It uses a sliding window to scan the video and multiple frame sequences in a sliding window form a candidate segment, so that after one scan, multiple candidate segments are generated. Each segment is regarded as an independent prediction unit. When multiple prediction results are generated for the same event, the segment with a probability value greater than a certain threshold is selected to enter the postprocessing stage. Through the sliding method, the entire input video can be uniformly processed and the context information of each time point can be preserved.

After candidate segments are generated, multiple frame sequences in each segment are input into 3D CNN to extract features. After BLSTM integration, the prediction result of this segment is generated, and the specific process is shown in Figure 6.

Among the existing algorithms for event detection or action detection using sliding windows, most of them treat the entire sequence as a whole and extract features for all frames. For short videos, better results can be achieved, while for football videos containing tens of thousands of frames, the amount of computation is greatly increased. Through analysis, it is found that there is little change between two adjacent frames. Therefore, in response to this problem, this section proposes to take one frame every two frames to form a frame sequence and then extract features. When a complete video is detected, the number of frames processed is reduced to one-half of the original, thus improving the computational efficiency.

After extracting the sequence features, it is necessary to use LSTM to further integrate the features. After the sequence features are integrated, the Softmax classifier is used to calculate the probability value of the segment corresponding to each category. The category with the highest probability is selected as the predicted category of the segment. The results output by the event detection model are fixed-size fragments that require a postprocessing stage to further determine the boundaries where the event occurred. Segments predicted to be nonevents in the output are first removed, and other segments are classified by event type. Then, according to the detection effect of different events, different probability thresholds are set, and all segments whose predicted probability value is greater than the threshold are respectively screened out. Finally, in the candidate segments of each category, the adjacent segments whose frame difference is less than 32 frames are merged to obtain a complete event.

### 4.3. Model Training

Football events often occur in specific scenes, which have a lot to do with the state of motion before and after it. Therefore, before training, the dataset is first augmented. When using sliding windows of different lengths to segment long videos, the event will be included in segments of different lengths, and start and end frames will be recorded. The intersection ratio of each segment and annotated event segments is calculated, and the segments with IoU > 0.65 are retained as positive samples to join the training set. Among them, the sliding window takes 32, 64, and 128 frames, and IoU is used to calculate the overlap between the candidate segment and the annotated segment. In addition, nonevent samples of different lengths are added as negative samples in the training set to improve the generalization ability of the model.

The event detection model is further trained on the basis of the classification model. Since the output category has more nonevent samples than the classification, when the parameters are initialized, the 3D CNN directly uses the corresponding parameter values that have been trained in the classification model as the initialization parameters. The BLSTM and Softmax classifiers use random initialization parameters, the initial learning rates are set to 0.001 and 0.01, respectively, and SGD is used to update the parameters. In 3D CNN, the kernel size is 3 × 3 × 3, the stride is 1, the pooling window size is 2 × 2 × 2, the stride is 2, and the dropout rate is 0.5. There are 256 hidden units in the hidden layer in BLSTM. When generating candidate segments, the sliding window size is 64 frames and the sliding step size is 16 frames. The sequence size used to extract features is 16 frames and the sliding step size is 8. In the training process, it is hoped to obtain a model with relatively small parameters, so that even if the input data has a certain deviation, it will not have a great impact on the results. To a certain extent, the phenomenon of overfitting is avoided. To this end, when setting the loss function, in addition to calculating the classification loss, L2 regularization is also added to limit certain parameters in the loss function to penalize the weights of unimportant features. The calculation method is as follows:

(3) $$\begin{array}{c} L=L_{0}+\frac{\lambda }{2m}\sum w^{2}, \end{array}$$

where *L*_0_ is the classification loss.

## 5. Experiment and Discussion

### 5.1. Dataset

The dataset used in this design is a self-made soccer match video dataset, with a total of 200 soccer match videos, including FIFA World Cup 2014, AFC Asian Cup 2015, and UEFA EURO 2016. Each game video is about 45 minutes long and has a frame rate of 25 fps. The dataset contains shots and events. Only the data part about the event is used in this design. Six types of events and corresponding playback shots are defined in the data set, and the types and quantities of each event are listed in Table 1.

Precision and recall are utilized as evaluation metrics in this work:

(4) $$\begin{array}{c} \text{Precision}=\frac{\text{Correct}}{\text{Correct}+\text{False}},\\ \text{recall}=\frac{\text{Correct}}{\text{Correct}+\text{Miss}}\text{.} \end{array}$$

### 5.2. Evaluation on Football Events Classification

First, the football event classification model proposed in this work is evaluated, and the experimental results are illustrated in Figure 7 and Table 2.

It can be seen from the detection results that better detection results can be achieved when performing classification prediction. Among them, the classification effect of corner kicks is the best, because corner kick events mainly occur in the four corner kick areas of the court, the positions are relatively fixed, and the rules are clear, which has more obvious distinguishing characteristics than other events. Accuracy and recall are also higher for yellow cards and fouls. Fouls usually cause players to fall to the ground, and the movement characteristics between players are relatively obvious. After a yellow card occurs after a foul, the referee shows the action of showing a yellow card continuously on the camera. The referee's jersey is different from the players and has a certain degree of recognition. Shooting incidents and goal-scoring incidents occurred in very similar scenes, and there were many misjudgments in the test. The goal event can be regarded as a kind of shooting event, and the only difference is the position of the ball. In football games, there are many players and complex sports scenes, which are prone to occlusion, so the position of the ball cannot be accurately determined. Coupled with the fact that the training samples of shooting events are far more than the training samples of goal events, it is easy to predict goal events as shooting events during classification. The classification effect of free kicks is poor, and there are two locations where free-kick events occur: inside the penalty area and outside the penalty area. When the incident occurs in the penalty area, it has obvious characteristics due to the certain rules of the positional arrangement of the players. When the incident occurs outside the penalty area, the scene has certain similarities with fouls, shots, etc., which will cause misjudgment.

This work uses the 3D CNN to extract features and verify the effectiveness of this strategy, and we compare it with the performance of the Inception v2 network. The experimental results are illustrated in Figure 8.

When using 3D CNN to extract features for event segments, the classification performance is better than using Inception v2 to extract single frame features. This is because 3D CNN better preserves the dynamic information between frames by extracting features from multiple frames at the same time. This dynamic information can effectively improve the effect of event classification.

This work uses the ReLU activation function to perform nonlinear activation of network features. To verify the effectiveness of this strategy, this work compares different activation functions. The experimental results are illustrated in Figure 9.

It is obvious that the football event classification performance when using the ReLU activation function is better than the sigmoid function and the tanh function.

As mentioned earlier, when training the event classification network, three different parameter tuning methods are proposed, which are named PA, PB, and PC, respectively. In order to verify the impact of different parameter tuning methods on network performance, a comparative experiment is carried out in this work, and the results are illustrated in Figure 10.

It can be seen that using the third parameter tuning method to fine-tune the parameters of all layers can achieve the best performance, which can constrain the network to learn more discriminative features.

### 5.3. Evaluation on Football Event Detection

To verify the performance of the football event detection network proposed in this work, different events are detected. The experimental results are listed in Table 3, and the training loss is illustrated in Figure 11.

It can be seen that the football event detection algorithm proposed in this work has obtained relatively good performance on different events. This proves the effectiveness and feasibility of this work.

As mentioned earlier, this work uses BLSTM to extract video features. To verify the effectiveness of this strategy, it is compared with the traditional LSTM method. The experimental results are illustrated in Figure 12.

It is obvious that higher football event detection performance can be obtained using BLSTM. This is because the BLSTM network is a bidirectional network that can extract more robust features.

As mentioned earlier, this work adopts the corresponding dataset expansion strategy (DE) when training the event detection network. To verify the effectiveness of this strategy, this work conducts comparative experiments to compare the event detection performance without DE and with DE, respectively. The experimental results are illustrated in Figure 13.

Obviously, after using the dataset expansion strategy, the precision and recall indicators of the event detection model have been improved to a certain extent. This proves the feasibility of using this strategy in this work.

Similarly, L2 regularization strategy is also used when optimizing the network. In order to verify the improvement of network performance by this strategy, corresponding comparative experiments are carried out. The experimental results are illustrated in Figure 14.

It is not difficult to see that after using the L2 regularization strategy, the optimization of the network is more effective. This improves the relative performance of football event detection.

Finally, this work presents a visual example of football video analysis, as shown in Figure 15.

## 6. Conclusion

In this work, a deep learning method is used to design a football event detection algorithm for football game video analysis. The algorithm can automatically detect and classify various events in football game videos. Among them, the three-dimensional convolutional network is used for feature extraction, which can process multiple frames of images at the same time, so as to retain relevant information between frames. It uses a bidirectional recurrent network to integrate features from both positive and negative directions to obtain past and future contextual information to improve the effect of event detection. The main content is divided into two parts: (1) classification of football events. The classification model employs the 3D CNN network and the Softmax classifier for feature extraction and predictive classification for event segments, respectively. According to the characteristics of the football game video, the model input is divided into a full-frame image and a central area of the frame, which are respectively put into 3D CNN to extract features, and feature fusion is performed. The Softmax classifier calculates the predicted value of each category for the event segment and selects the one with the largest predicted value as the predicted category of the event. (2) Football event detection: the event detection model is based on the classification model by adding the BLSTM structure to better obtain dynamic information between multiple frame sequences. During training, the dataset is expanded first, and then the event detection model is optimized using the SGD algorithm. During testing, a sliding window is used to segment the video, input each segment into the model, and calculate the predicted values for all the corresponding categories. Through filtering and merging, the start and end boundaries of events are further confirmed, and category labels are generated. To verify the validity and correctness of proposed method, comprehensive and systematic experiments are carried out, and the model is analyzed from different aspects. The experimental results confirm the feasibility of this work.

## Figures and Tables

**Figure 1:** The football event detection.

**Figure 2:** The structure of inception.

**Figure 3:** The event classification model.

**Figure 4:** The structure of 3D CNN.

**Figure 5:** Football event detection process.

**Figure 6:** Event fragment prediction process.

**Figure 7:** The training loss on football events classification.

**Figure 8:** Comparison of Inception v2 and 3D CNN.

**Figure 9:** Comparison of different activation functions.

**Figure 10:** Comparison of different tuning methods.

**Figure 11:** The training loss on football event detection.

**Figure 12:** Comparison of BLSTM and LSTM.

**Figure 13:** Evaluation on dataset expansion strategy.

**Figure 14:** Evaluation on L2 regularization strategy.

**Figure 15:** The visual example of football video analysis.

**Table 1:** Distribution of various events.

Event	Training set	Test set
Shot	1350	611
Corner kick	691	276
Free kick	652	259
Yellow card	225	152
Foul	1683	690
Goal	155	72

**Table 2:** Football event classification results.

Event	Precision	Recall
Shot	78.8	84.9
Corner kick	90.1	95.6
Free kick	78.9	63.8
Yellow card	97.9	81.2
Foul	87.1	89.9
Goal	30.6	14.9
Average	77.2	71.7

**Table 3:** Football event detection results.

Event	Precision	Recall
Shot	19.7	85.1
Corner kick	39.2	86.9
Free kick	18.2	45.6
Yellow card	10.5	45.2
Foul	12.3	55.7
Goal	18.5	6.7
Average	19.7	54.2

## Data Availability

The datasets used during the current study are available from the corresponding author on reasonable request.
